This article has been retracted.

# Design of the Exercise Load Data Monitoring System for Exercise Training Based on the Neural Network

**DOI:** 10.1155/2021/7340140

**Published:** 2021-09-24

**Authors:** Panlong Qin, Wei Feng

**Affiliations:** Department of Physical Education, Hebei Academy of Fine Arts, Hebei,050700, China

## Abstract

In order to monitor the sports load data of athletes in sports training, this paper studies the methods and systems of sports load monitoring and fatigue warning based on neural network technology. In this paper, the neural network parallel optimization algorithm based on big data is used to accurately estimate the motion load and intensity according to the determined motion mode and acceleration data, so as to realize the real-time monitoring of the exercise training. The results show that the value of *η* is usually small to ensure that the weight correction can truly follow the direction of the gradient descent. In this paper, 176 samples were extracted from the monitoring data collected by the “National Tennis Team Information Platform,” 160 of which were selected as training samples and the other 16 as test samples. Ant colony size *M* = 20. The minimum value *W*_min_ of the weight interval is −2, and the maximum value *W*_max_ is 2. The maximum number of iterations is set to 200. *σ* = 1; that is, only one optimal solution is retained. The domain is divided into 60 parts evenly; that is, *r* = 60. Generally, *η* can be taken as any number [28] between [10-3, 10], but the value is usually small to ensure that the weight correction can truly follow the direction of the gradient descent. In this paper, the value is 0.003. In the early warning stage of exercise fatigue, reasonable measurement units of exercise fatigue time were divided according to the characteristics of different exercise items. It is proved that the Bayesian classification algorithm can effectively avoid the sports injury caused by overtraining by warning the fatigue and preventing the sports injury caused by overtraining.

## 1. Introduction

Artificial neural network (ANN) is a kind of nonlinear dynamic system, which is borrowed from the development of biological neural network [1], the new intelligent information processing system. With its unique information processing methods, ANN has been widely used in various fields, such as industrial production monitoring, classification, prediction and forecasting, analysis and processing, auxiliary diagnosis of diseases, environmental pollution, and purification prediction. BP neural network is one of the representative neural network models and has been widely used. However, BP algorithm has some defects, such as low efficiency, slow convergence speed, and being easy to fall into local minimum, which restrict the application of BP network in various fields [2]. Ant Colony Optimization (ACO) is a novel bionic evolutionary algorithm, which shows excellent performance and great development potential in solving complex optimization problems, especially discrete optimization problems. ACO, as a global optimization heuristic algorithm, is used to train the weight of neural network, which can avoid the defect of BP neural network. Nowadays, the competition of sports science and technology is increasingly fierce [3]. It is necessary to have scientific training methods and means in order to improve sports performance. Sports competition is a big competition of science and technology. The guiding ideology of implementing competitive sports science and technology work is to carry out the thought that science and technology is the first productive force, carry out the strategy of “invigorating sports through science and education,” and perfect the management system and movement mechanism that sports training and sports science and technology are closely combined [4]. Our research focuses on the actual needs in training, aiming at the key problems in training practice, to carry out scientific research and public relations, and strengthen technical innovation. To promote the scientific sports training, give full play to the leading role of science and technology and improve the sports skills of our athletes and the competitive strength in the world competition, for our athletes in the 2008 Olympic Games to get good results to win the gold medal to make contributions [5].

## 2. Literature Review

In this paper, the detection data of physiological and biochemical indexes of national athletes were taken as training samples, and the ACO-BP algorithm was adopted to integrate ACO and BP algorithm to complete the neural network training [6, 7]. The ant colony neural network prediction model was established for sports load, and the corresponding relationship between physiological and biochemical indexes in sports and training load was obtained. Firstly, ACO is used to optimize the neural network weights as a whole to overcome the shortage of BP algorithm which is easy to fall into local optimum [8, 9]. Then taking the better weight as the initial value, BP algorithm is used to do further optimization, to overcome the shortcomings of a single ACO training network with long time and low precision [10–12].

The research continues; Jeon and Kim used artificial intelligence and expert system design principle, and the method of simulated medical expert diagnosis, treatment of disease thinking process, and compiled computer program can help doctors to solve complex medical problem, as the doctor concluded that it is an important auxiliary tool for the treatment of disease and prognosis. Medical expert system is an important application of artificial intelligence in medicine. It is a collection of knowledge, computer technology, network technology, communication technology, database technology, and medical science. The development of medical expert system has become an important topic in modern medicine [13]. Cavina et al. designed a multiprotocol recognition system based on BP artificial neural network. The specific research contents of this paper include the design of multiprotocol recognition eigenvalue, the data of a certain length of frame head is taken as the eigencode, and the eigenvalue is obtained after normalized processing. The selection of multiprotocol learning algorithm, simulation analysis, and comparison of several BP neural network algorithm is according to the convergence rate and recognition rate of conjugate gradient descent method as the multiprotocol recognition system BP neural network identification algorithm. As per the establishment of multiprotocol recognition network, through simulation, according to the recognition rate, the maximum number of hidden layer of BP neural network suitable for the multiprotocol recognition system in this paper is 9. The design of multiprotocol identification system, aiming at the characteristic of the relatively fixed address of the monitoring terminal in power transmission, adopts the measures of establishing identification table in the system and judging whether the data frame sent by the terminal address has been sent before identification, so as to improve the real-time performance of the identification system [14]. Zhou et al. designed a neural network compensator based on the nonlinear error of the motion control system of the image measuring instrument. The neural network simulator and compensator of nonlinear servo motor are trained by the data of input and output of servo motor. The designed neural network compensator is applied to the high precision positioning system of motion control, which makes the control system show good control performance. Simulation results show that the controller is effective [15]. With the continuous maturity and development of artificial neural network technology, the intelligent characteristics and capabilities of neural network are increasingly expanded in its application fields. Many problems that cannot be solved by traditional information processing methods have achieved good results after using neural network, and especially in the engineering field it has been widely used. With the continuous development of neural network theory itself and related theories and technologies, the application of artificial neural network will be more in depth and extensive.

In this paper, the test data of Chinese athletes' physiological and biochemical indexes are taken as training samples, and the ACO and BP algorithm are combined to complete the neural network training method, namely ACO-BP algorithm, to establish the ant colony neural network prediction model for the exercise load and obtain the corresponding relationship between the physiological and biochemical indexes and the training load during the exercise. Firstly, ACO is used to optimize the weight of the neural network globally to overcome the shortcoming of BP algorithm which is easy to fall into local optimal. Then, with the optimal weight as the initial value, BP algorithm is used to do further optimization, so as to overcome the disadvantages of a single ACO training network such as long time and low accuracy.

## 3. Research Methods

Theoretical analysis proves that a feedforward net with a single hidden layer can map all continuous functions only when learning. Two hidden layers are required when the function is discontinuous. Increasing the number of hidden layers can improve the nonlinear mapping ability of BP network, but when the number of hidden layers exceeds a certain value, the performance of BP network will decline. In 1998, Hecht-Nielson proved that a continuous function in any closed interval can be approximated by a BP network with a hidden layer. Therefore, this paper will adopt a three-layer BP network with a hidden layer, namely, R-N-1. Neural network structure model is where *n* is the number of input nodes, *r* is the number of hidden nodes, and the number of output nodes is 1. The number of neurons in the input layer of the neural network is determined by the influencing factors [16, 17]. In this paper, the physiological and biochemical indexes which can obviously reflect the physiological function and the professional training years are taken as the influencing factors. The number of nodes in the output layer is set as 1, and the value range is [−1, 1], which is used as the quantified value to measure the load. The closer the value is to 1, the smaller the load is, and vice versa.

The role of hidden layer nodes is to extract and store the inherent rules from the samples. Each hidden layer node has several weights, and each weight is a parameter to enhance the mapping ability of the network. If the number of hidden nodes is too small, the network's ability to obtain information from the sample is poor, which is not enough to summarize and reflect the sample rule of the training sample. If the number of hidden nodes is too large, it may also learn to remember the irregular content of the sample, such as noise, which reduces the generalization ability.

Generally, the following empirical formula can be used for the number of hidden layer nodes in three-layer forward network:

(1) $$\begin{array}{c} m=\sqrt{n+1}+a,\\ m=\log\;2^{n},\\ m=\sqrt{nl}. \end{array}$$

*M* is the number of nodes in the hidden layer, N is the number of nodes in the input layer, *L* is the number of nodes in the output layer, and *α* is a constant between 1 and 10. In this paper, the number of hidden layer nodes is determined according to equation (1). To sum up, the BP neural network adopted in this paper is shown in Figure 1.

### 3.1. Processing of Sample Data

Tennis sport has the longer game time, the intensity of the intermittent type, short smell, and explosive force action composition. Tennis is more and more towards the strength and speed against the direction of development; the physical requirements are very high. With the increase of professional training years, various functions of the body will change, and the ability to adapt to the load will also change. Athletes with short training years can bear less amount of exercise than those with long training years. The same amount of exercise may be a large exercise load for young players. Therefore, the professional training years can be used as an important influencing factor of load forecasting to improve the accuracy of assessment ability.

The training samples used in the experiment are from the tennis team sports collected by the “National Tennis Team Information Platform” physiological and biochemical indexes monitoring information of the mobilized competition and daily training. Due to the size of the original test data, in order to avoid the difference of physical meaning and unit of input vector on the network model, the difference of bit is obvious. Before the training of neural network, the training samples need to be processed in advance, that is, normalized processing [18, 19]. In order to train the function better, we also can avoid the network failure caused by being too large. The numbers are collected in this article. The data are mapped between [−1, 1] and normalized, so that the normalized input and target data are subject to normal distribution; i.e.,

(2) $$\begin{array}{c} \left[pn,\text{mean}p,\text{std}p\right]=\text{prestd}\left(p\right),\; \end{array}$$

where *pn* is the input direction after vectorization, *p* is a group of collected data (vector), and mean*p* is the input direction after vectorization. Enter the mean value of the vector, and STDP is the deviation of the input vector. The algorithm executed is

(3) $$\begin{array}{c} pn=\frac{\left(p-\text{mean}p\right)}{\text{std}p}. \end{array}$$

As physiological and biochemical indexes, some indexes are correlated. Through the principal component analysis of standardized data, the redundant components of sample data can be eliminated; that is, the components that contribute little to the overall change of the data set, so as to reduce the data dimension. The processing function of MATLAB is

(4) $$\begin{array}{c} \left[P\text{trans},\text{TransMat}\right]=\text{prep}ca\left(pn,0.02\right); \end{array}$$

where 0.02, the second parameter in the prep*ca* function, indicates that the main element is an element whose square deviation from the mean is greater than 2% of the variance of the vector. TransMat is a change matrix with major elements.

In this paper, the blood data and urine data were analyzed by principal component analysis. Through the analysis and processing of a group of processed blood test data and urine data of national tennis team players, the urine sample data were changed from the original 9. The dimension (8 dimensions of urine index and professional training years) was reduced to 6, and the data of blood data were reduced to 13 from 15 (14 dimensions of blood index and professional training years).

### 3.2. Basic Steps

In the case that the structure of the neural network has been determined, the basic steps of training the neural network by the ACO-BP method are as follows:

Step 1: initialize:
The weights of all the weights of the interval [*W*_min_ and *W*_max_] are evenly divided into *r* subregions. Each region that the points on the boundary is the value of an alternative for each parameter setting up a list of pheromones as shown in Table 1. At the initial moment, set each point to have the same amount of pheromone tau 0, pheromone volatilization coefficients rho, and time *t,* and the number of loop NC is zero. Set the maximum number of loops of the ending condition, MAXNC.
Step 2: release all *M* ants. Ant *K* uses the following probability formula as a path selection rule. That is, select an element in each set Ipi(1≤ *I* ≤ *m*).
  (5) $$\begin{array}{c} p_{k}\left(i\right)=\frac{\tau \left(i\right)}{\sum_{1\leq j\leq m}\tau \left(i\right)}. \end{array}$$
To record the label of the point passed by the ant, a value is selected for the weight and recorded in K. After the ant selects the values for all the weight parameters, the ant completes a traversal, and all the values it chooses to record constitute all the parameters of the neural network.
Step 3: repeat Step 2 until all the ants reach the food source.
Step 4: let *T* ← + *M*, NC ← NC + 1. Use the weight parameters selected by each ant to calculate the output results of the neural network and the error *E*, record the weight of *σ* group with small error and the current optimal solution Emin, and compare the size of Emin and E0. If Emin ≤ *E*0, go to Step 8; otherwise, go to Step 5.
Step 5: update the pheromone of each element according to the pheromone regulation rules below. Pheromone regulation: as time goes by, the pheromone that was left behind gradually fades away. The volatility coefficient *ρ* represents the persistence of the pheromone, and 1−*ρ* represents the vanishing degree of the pheromone. After *n* time units, the ants travel from the nest to the food source, and the pheromones along each path are adjusted according to the following formula:
  (6) $$\begin{array}{c} \tau_{j}\left(I_{pi}\right)\left(t+m\right)=p\tau_{j}\left(I_{Pi}\right)\left(t\right)+\Delta \tau_{j}\left(I_{pi}\right),\\ \Delta \tau_{j}^{k}\left(I_{pi}\right)=\left\{\begin{array}{c} \frac{Q}{e^{k}},\\ 0, \end{array}\right) \end{array}$$
where *Q* is a constant, used to adjust the pheromone adjustment speed. *e*^*k*^ is the output error when a set of weights selected by the KTH ant is taken as the weights of the neural network and is defined as *e*^*k*^=|*o* − *o*_*q*_|, where *o* and*o*_*q*_ are the actual and expected outputs of the neural network. As you can see, the smaller the error, the larger the corresponding pheromone increase.
Step 7: the neural network is further trained by BP algorithm, the best weights of *σ* group found by ANT colony algorithm are taken as the initial weights of BP algorithm, the error between network output and actual output is calculated, and the error is propagated one-way from the output layer to the input layer to adjust the weights. Repeat the process until the stop conditions are met.
Step 8: use validation samples to test the generalization ability of the trained neural network. If the validation error meets the requirements, quit the program. Otherwise, go to Step 1 and start training again.

## 4. Result Analysis

In order to verify the network model, the author has done a lot of computer simulation experiments. In women's team sports, as an example, the blood index data of the team members were collected from the monitoring data collected by the “National Tennis Team Information Platform.” 176 samples were taken, and 160 of them were selected as training samples and the other 16 were selected as test samples. Ant colony size *M* = 20. The minimum value of the weight interval *W*_min_ is −2, and the maximum value *W*_max_ is 2. The maximum number of iterations is set to 200. *σ* = 1; that is, only one optimal solution is retained. The domain is evenly divided into 60 parts; that is, *r* = 60; *η* can generally take any number between [10-3, 10], but it usually takes a small value to ensure that the weight correction can really descend along the direction of the gradient. In this paper, the value is 0.003. The specific parameter settings of the network are shown in Table 2.

According to the actual situation of the national tennis team and the need of preparing for the Olympic Games, the national tennis team information platform is designed and developed with Delphi7.0 development tool and SQL Server2000 database. The information platform includes athletes' basic information, athletes' training and competition information data, image and video analysis and training monitoring data, which is a set of analysis and management system for tennis. It mainly stores the basic information of Chinese tennis players, athletes' injuries and rehabilitation, nutritional recovery information, athletes' special energy, physiology and biochemistry, training load, training method, training course content, training effect, competition process, competition results, and other training match information data. From the perspective of function, it mainly includes data management, video image management, and data analysis.

The output results corresponding to the samples were jointly determined by experts, team doctors, and other people in combination with the corresponding training plans and athletes' performance at that time. We use minus 1 for body function. Poor athletes cannot adapt to the current training plan and should immediately adjust the amount of training. Let us denote the athlete by 0. Being able to adapt to the current training plan, exercise amount is appropriate and can maintain the training plan for training; 1 indicates that the body function is in a completely normal state, the athletes can fully adapt to the current amount of exercise, and can appropriately increase the amount of training to improve the training effect. The test results obtained through the simulation test are listed in Table 3.

From the above experimental results, the following conclusions can be drawn: the three-layer front is based on ant colony optimization algorithm presented in this paper. Based on the training model of feedback neural network (BP neural network), a new network training algorithm is established. The experimental results are analyzed and compared with the standard BP algorithm and the improved BP algorithm with momentum term, ACO-BP. The algorithm has a fast convergence speed and can achieve a smaller value of mean square error. Therefore, the convergence process of this method has obvious advantages and stability.

## 5. Summary of This Paper

In order to monitor the sports load data of athletes in sports training, this paper studies the methods and systems of sports load monitoring and fatigue warning based on neural network technology. In this paper, the neural network parallel optimization algorithm based on big data is used to accurately estimate the motion load and intensity according to the determined motion mode and acceleration data, so as to realize the real-time monitoring of the exercise training. The results show that the value of *η* is usually small to ensure that the weight correction can truly follow the direction of gradient descent. In this paper, 176 samples were extracted from the monitoring data collected by the “National Tennis Team Information Platform”, 160 of which were selected as training samples and the other 16 as test samples. Ant colony size *M* = 20. The minimum value *W*_min_ of the weight interval is −2, and the maximum value *W*_max_ is 2. The maximum number of iterations is set to 200. *σ* = 1; that is, only one optimal solution is retained. Divide the domain into 60 parts evenly; that is, *r* = 60. Generally, *η* can be taken as any number [28] between [10-3, 10], but the value is usually small to ensure that the weight correction can truly follow the direction of gradient descent. In this paper, the value is 0.003. In the early warning stage of exercise fatigue, reasonable measurement units of exercise fatigue time were divided according to the characteristics of different exercise items. It is proved that the Bayesian classification algorithm can effectively avoid the sports injury caused by overtraining by warning the fatigue and preventing the sports injury caused by overtraining. The research of this paper is a preliminary study, combined with ability and the limitation of technical conditions. There are a lot of improvement, mainly having the following several aspects: (1) the ant colony algorithm is a new bionic algorithm. Now still not mature, the parameters of the ant colony algorithm selection theoretical guidance remain to be further strengthened, because it directly relates to the parameter selection of application effect of the algorithm. (2) The ant colony algorithm is further improved to increase the convergence of the improved ant colony algorithm to meet the needs of large-scale network. (3) Integrate qualitative and quantitative problems, and quantify fuzzy concepts, so as to better meet the needs of users.

## Figures and Tables

**Figure 1:** BP network structure.

**Table 1:** Pheromone table of weights.

Label	1	2	...	*r* + 1
Divide the scale	*a*1	*a*2	...	*ar* + 1
The pheromone values	(1)	(2)	...	(*r* + 1)

**Table 2:** ACO-BP and BPNN parameter settings.

The name of the	*M*	*W*_min_	*W*_max_	*Q*	*r*	NACO		NBP	EO
ACO-BP	20	−2	2	0.005	60	200	0.003	12000	0.005
BPNN		−0.1	0.1				0.003	20000	0.005

**Table 3:** Comparison of simulation test results.

The experimental method	The mean square error of the *N*th iteration		
	*N* = 100	*N* = 500	*N* = 1000
Standard BP algorithm	0.00977462	0.0063423	0.00429856
BP algorithm for adding the momentum term	0.00868283	0.00416346	0.000683606
ACO-BP algorithm	0.0071246	0.00198015	8.9427*e* − 5

## Data Availability

The data used to support the findings of this study are available from the corresponding author upon request.
